This article has been retracted.

# Free Triiodothyronine Is Independently Associated with Nonalcoholic Fatty Liver Disease in Hospitalized Type 2 Diabetes Mellitus Patients

**DOI:** 10.1155/2021/8868339

**Published:** 2021-01-19

**Authors:** Rou Shi, Chunwen Lin, Yaping Hong, Xiaoying Xia, Yingjian Chen, Shu Li, Liangchang Xiu

**Affiliations:** ^1^Department of Epidemiology and Medical Statistics, School of Public Health, Guangdong Medical University, Dongguan, Guangdong 523808, China; ^2^Huizhou Municipal Central Hospital, Huizhou, Guangdong 516008, China; ^3^Shenzhen Longhua District People's Hospital, Guangdong 518000, China

## Abstract

**Objective:**

Free triiodothyronine (FT3) is an independent risk factor for nonalcoholic fatty liver disease (NAFLD) in patients with euthyroid. However, whether FT3 has an independent effect on NAFLD in a population of type 2 diabetes remains unknown. The purpose of this study was to identify the potential role of FT3 in NAFLD with T2DM.

**Design:**

A cross-sectional study. *Patient*. A total of 859 T2DM patients who met the inclusion criteria were included. There were 506 T2DM patients without NAFLD and 353 T2DM patients with NAFLD.

**Methods:**

The independent samples *t*-test or Wilcoxon rank sum test were used for continuous variables of different distribution types, while the chi-square test was used for categorical variables. Pearson correlation analysis and linear regression were used to analyze the correlation between FT3 and clinical measurements and biochemical indicators. Multivariate logistic regression analysis was used to determine independent predictors.

**Results:**

Patients with NAFLD had higher BMI, SBP, and DBP, longer duration of T2DM, and higher islet function index, blood glucose index, liver function index, renal function index, blood lipid index, and FT3. We also found that FT3 was affected by other five indicators, including ALT, CR, GGT, TC, and LDL-C only in the NAFLD group but not in the non-NAFLD group. FT3 was significantly associated with NAFLD in T2DM patients, and the prevalence of NAFLD increased gradually from the lowest FT3 tertile to the highest FT3 tertile (*P* for trend < 0.001).

**Conclusion:**

FT3 is independently associated with NAFLD in hospitalized T2DM patients after rigorous adjustment for various metabolic parameters.

## 1. Introduction

Growing evidence indicates that the prevalence of nonalcoholic fatty liver disease (NAFLD) in type 2 diabetes mellitus (T2DM) has increased significantly [1, 2]. A large-scale meta-analysis shows that the pooled prevalence of NAFLD in T2DM patients is about 60% [3]. NAFLD and T2DM often collaborate to cause adverse consequences, not only increasing the risk of diabetic complications, including macrovascular and microvascular complications, but also increasing the risk of more severe NAFLD, such as cirrhosis [4].

Free triiodothyronine (FT3) is essential for the growth, development, and metabolism of tissues and organs. Many studies have shown a positive association of FT3 levels with NAFLD among the euthyroid population [5, 6]. A 2.2-year follow-up study revealed that the increase in FT3 levels was correlated with the development of NAFLD in women with normal thyroid function [6]. The association between FT3 and adverse metabolism (including hyperglycemia, mixed hyperlipidemia, hypertension, and obesity) has been widely recognized [7, 8]. Recent reports have suggested that FT3 levels were related to the progression of insulin resistance, and low FT3 was significantly related to the decrease in HOMA-IR (adjusted coefficient = −1.151, 95% CI: −1.952, −0.350) in nondiabetic individuals [7, 8]. It is known that insulin resistance, obesity, and mixed hyperlipidemia are common risk factors for NAFLD and T2DM [9, 10]. However, whether FT3 is associated with NAFLD in patients with T2DM and whether it can be used as an indicator of risk for NAFLD in patients with T2DM remain unknown.

In this survey, we enrolled 859 T2DM patients. Clinical characteristics of T2DM patients with and without NAFLD were described, and the difference of biochemical indicators between two groups was compared. Then, the relationship between FT3 and biochemical indicators was analyzed, and four models were constructed to explore the association between FT3 and NAFLD in T2DM patients after adjusting for other factors. Discovery of this study can provide evidence to further study the mechanism and therapeutic targets of FT3 in NAFLD.

## 2. Patients and Methods

### 2.1. Study Design and Participants

We collected clinical data of 936 T2DM inpatients from January 2015 to October 2019 at Shenzhen Longhua Central Hospital. The patients were included in this study according to the following criteria: (1) T2DM was diagnosed using 1999 WHO criteria; (2) there is no history of drinking or having abstained from alcohol; (3) there is no other liver-derived fatty liver disease induction, e.g., viral hepatitis, drug-induced hepatitis, or autoimmune liver disease; (4) there are no serious complications of diabetes, such as hyperglycemia and hypertonic state, and patients with severe hypoglycemia; and (5) liver b-ultrasounds were performed in all inpatients, the liver ultrasound imaging features are consistent with a diffuse fatty liver, and the kidney ultrasound imaging features are used as a reference. According to the inclusion criteria, a total of 77 people were excluded (Figure 1). Eventually, 859 patients were included in the research. Among them, 353 (41.1%) had T2DM with NAFLD and 506 (58.9%) had T2DM without NAFLD.

### 2.2. Data Collection

The basic information and measurement indicators of all participants were inquired and measured by a professional nurse on the day when the patient entered the hospital. The basic information included gender, age, occupation, T2DM duration, address, smoking and drinking history, and T2DM family history. Measurement indicators included height, weight, hip circumference (HC), abdominal circumference (AC), blood pressure (BP), and admission blood glucose (ABG).

27 biochemical indicators were also tested for all participants in our hospital laboratory. Fasting (at least 8 hours of fasting) venous blood samples were collected to measure 19 biochemical indicators: fasting blood glucose (FBG), fasting insulin (FINS), glycated hemoglobin (HbA1c), thyroid-stimulating hormone (TSH), free triiodothyronine (FT3), free four iodothyronine (FT4), alanine transferase (ALT), aspartate aminotransferase (AST), glutamyl transpeptidase (GGT), urea nitrogen (UN), creatinine (CR), uric acid (UA), triglycerides (TG), total cholesterol (TC), high-density lipoprotein cholesterol (HDL-C), low-density lipoprotein cholesterol (LDL-C), C-reactive protein (CRP), D-dimer (DDi), and homocysteine (HCY). One hour (1 h) and two hours (2 h) after a 75 g oral glucose load, venous blood samples were collected to detect 1 h blood glucose (1hBG), 1 h insulin (1hINS), 1 h C peptide (1h-CP), 2 h blood glucose (2hBG), 2 h insulin (2hINS), and 2 h C peptide (2h-CP). In addition, 24 h total urine was also collected to measure 24-hour urine protein quantification (24h-UTP) and 24-hour urine albumin quantification (24h-ABL).

It is widely accepted that insulin resistance (IR) is closely related to NAFLD and T2DM. So, we calculated indicators of insulin resistance and islet *β*-cell function. The calculation formula is as follows: HOMA IR = fasting plasma glucose (mmol/L) × fasting plasma insulin (*μ*U/mL)/22.5; HOMA-*β* is as follows: HOMA‐*β* = 20 × fasting insulin level (FINS, mIU/L)/(fasting blood glucose level (FPG, mmol/L) − 3.5) (%). In order to better evaluate the kidney function index, we calculated the glomerular filtration rate (GFR). According to different genders, male GFR = [(140 − age) × weight (kg)]/[0.818 × blood creatinine (Scr, *μ*mol/L)] and female GFR = [(140 − age) × weight (kg)]/[0.818 × blood creatinine (Scr, *μ*mol/L)] × 0.85.

### 2.3. Statistical Analysis

All data were analyzed using IBM SPSS Statistics 25.0. The data of continuous variables are expressed as *x* ± *s* or median (interquartile range), and the categorical variables are expressed as the number of cases (*n*) or percentage (%). The independent samples *t*-test or Wilcoxon rank sum test were used for continuous variables of different distribution types, while the chi-square test was used for categorical variables. Pearson correlation analysis and multiple linear regression were used to analyze the correlation between FT3 and 29 variables to provide a basis for building models. Then, multivariate logistic regression analysis was performed on the important variables in the univariate analysis in four models to identify independent factors related to NAFLD. Finally, we perform FT3 tertiles (tertile 1: FT3 < 4.19; tertile 2: 4.19 ≤ FT3 < 4.87; and tertile 3: FT3 ≥ 4.87), use the chi-square test to compare the differences between groups, and evaluate the trend of FT3 level and NAFLD prevalence. *P* < 0.05 was considered statistically significant.

Four models are used for multiple logistic regression analysis: model 1 (adjusted for age, gender, T2DM duration, BMI, SBP, DBP, smoking history, TSH, and FT4), model 2 (adding F-CP, 2h-CP, AbG, FbG, 2hbG, HOMA-IR, and HbA1c on the basis of model 1), model 3 (adding urea, CR, UA, and eGFR to model 2), and model 4 (adding ALT, AST, GGT, TC, TG, HDL-C, and LDL-C to model 3). *P* < 0.05 was considered statistically significant.

### 2.4. Patient and Public Involvement

No patient was involved.

## 3. Results

### 3.1. Clinical Characteristics of Participants

For 353 T2DM patients with NAFLD, the NAFLD group, the mean age was 49.51 ± 12.22 years and 61.5% was male. For the other group, the non-NAFLD group (506 T2DM without NAFLD), the mean age was 51.41 ± 13.80 years and 63.0% was male. BMI, AC, HC, SBP, DBP, duration of T2DM, and reason for hospitalization were significantly different between the two groups. Patients with NAFLD had higher BMI, SBP, and DBP, larger AC and HC, and longer duration of T2DM. See Table 1 for details.

From Table 2, we observed that 19 indicators had significant differences between the two groups (*P* < 0.05). Compared to the non-NAFLD group, NAFLD group patients had higher islet function index (FINS, FCP, 1h-CP, and 2h-CP), blood glucose index (FBG, 1hBG and 2hBG), liver function index (AST, ALT and GGT), renal function index (CR, UA, and GFR), and blood lipid index (TC and TG) and had lower ABG, UN, and DDi. In terms of thyroid function, FT3 was higher in NAFLD patients, but there was no significant difference in TSH and FT4 between the two groups.

### 3.2. Correlations between FT3 and Clinical Parameters

Pearson correlation analysis showed that FT3 was significantly negatively correlated with age, ABG, HbA1c, TSH, and UN in the two groups. Compared with the non-NAFLD group, the correlations between FT3 and age, ABG, and HbA1c were more close (correlation coefficient = −0.342, -0.204, and -0.173, respectively) in the NAFLD group. It is worth noting that in the NAFLD group, FT3 was significantly positively correlated with ALT, LDL-C, and GFR and significantly negatively correlated with CR and HDL-C. However, there was no correlation between FT3 and these indicators in the non-NAFLD group (Table 3).

Multiple linear regression analysis showed that FT3 levels were affected by five indicators, including age, ABG, HbA1c, LDL-C, TSH, and LDL-C in the two groups. Compared with the non-NAFLD group, these five indicators have a greater impact on FT3 levels in the NAFLD group (age (*b* = −0.023), ABG (*b* = −0.3), HbA1c (*b* = −0.075), LDL-C (*b* = 0.187), and TSH (*b* = −0.022)). Take HbA1c as an example; with all other factors being held constant, with the increase in HbA1c, the FT3 level decreased. Every 1% increase in HbA1c will cause the level of FT3 to decrease by 0.069 pmol/L in the non-NAFLD group but 0.075 pmol/L in the NAFLD group. We also found that FT3 was affected by other five indicators, including ALT, CR, GGT, TC, and LDL-C only in the NAFLD group but not in the non-NAFLD group (Table 4).

### 3.3. Multiple Logistic Regression Models

After adjusting for gender, age, T2DM duration, BMI, SBP, DBP, smoking history, TS, and FT4, FT3 was significantly associated with the prevalence of NAFLD (model 1, OR = 1.288, 95% CI 1.062-1.562, *P* < 0.05). Interestingly, by adding F-CP, 2h-CP, ABG, FBG, 2hBG, HOMA-IR, and HbA1c on the basis of model 1, FT3 showed significant associations with the prevalence of NAFLD (model 2, OR = 1.286, 95% CI 1.006-1.644, *P* < 0.05), and it was still statistically significant after further adjustment for urea, CR, UA, and eGFR (model 3, OR = 1.367, 95% CI 1.068-1.751, *P* < 0.05). In model 4, we added ALT, AST, GGT, TC, HDL-C, LDL-C, and TG on the basis of model 3, and the probability that a patient had NAFLD increased as FT3 level elevated (OR = 1.301, 95% CI 1.028-1.645, *P* < 0.05). See Table 5 for details.

We conducted multiple regression analysis of variables in model 4 to screen variables with statistical significance. Then, we used the logistic proportional hazards regression model to construct a nomogram containing variables filtered from model 4 (age, BMI, DBP, FT4, FT3, FCP, CR, and hbG). From Figure 2, we can predict that when other influencing factors remain unchanged, the risk of disease will increase with the increase in FT3 level. See Figure 2 for details.

The corresponding line segment of each variable is marked with a scale, which represents the value range of this variable, while the length of the line segment reflects the contribution of this factor to the ending event. The points in the figure represent the individual score corresponding to each variable under different values. The total points in the figure represent the total score of the corresponding single score after all variables are evaluated. Based on the total score, we can predict the risk of the disease.

### 3.4. Prevalence of NAFLD in T2DM Patients Based on FT3 Tertiles

In Figure 3, we found that the prevalence of NAFLD increased gradually from the lowest FT3 tertile to the highest FT3 tertile (32.1%, 41.3%, and 49.4%). As the FT3 tertile increases, the prevalence of NAFLD gradually increases (*P* for trend < 0.001). However, compared with tertile 1, tertile 2 (*P* = 0.026) and tertile 3 (*P* < 0.001) significantly increased the prevalence of NAFLD.

## 4. Discussion

Many studies have proven that FT3 was independently positively related to the risk of NAFLD in euthyroid subjects [11, 12]. In this study, we described the clinical characteristics and compared the differences of biochemical parameters between the two groups in 859 T2DM patients. Then, we analyzed the correlation between FT3 and biochemical parameters and the association between FT3 and NAFLD prevalence. The study led to a key conclusion that FT3 was an independent risk factor for NAFLD in T2DM patients.

Among nondiabetic populations with euthyroid, patients in the NAFLD group were older compared to patients in the non-NAFLD group [5, 6]. However, we found that NAFLD patients were younger and had shorter T2DM duration in the T2DM population. A recent study based on the T2DM population also confirmed our results [13]. Patients in the non-NAFLD group were older, and T2DM duration lasted longer. This phenomenon may be related to these T2DM patients with long-term oral hypoglycemic, lipid-lowering, and other drugs that regulate metabolism. A recent study showed that many hypoglycemic drugs have shown the benefit of improving metabolic parameters and reducing liver lipid accumulation in NAFLD patients [13]. It has been found that metformin is important to improve abnormal metabolic parameters in patients with T2DM and NAFLD [14].

Univariate analysis showed that there were significant differences in 19 biochemical indexes among different groups, including FT3. A study based on the T2DM population shows that 10 biochemical indicators (FINS, 2hBG, TC, TG, AST, ALT, GGT, UA, eGFR, and HOMA-IR) are significantly different between the non-NAFLD group and NAFLD group [13]. These differences are in line with our findings. However, our research also found that C-peptide (F-CP, 1h-CP, and 2-CP), renal function indicators (UN, CR), and DDi were also significantly different in the two groups. Early renal impairment and other chronic kidney diseases can present with NAFLD [15]. US and Chinese studies have shown a significant association between C-peptide and the presence of NAFLD [16, 17].

We found that in the NAFLD group, FT3 was significantly correlated with 10 indicators: age, ABG, HbA1c, HDL-C, LDL-C, ALT, TSH, UN, GFR, and CR. A study based on the T2DM population also found similar results to ours [7]. After adjusting for age, BMI, T2DM duration, TSH, FT4, and HbA1c, FT3 level is still affected by 6 indicators: ABG, TC, LDL-C, ALT, GGT, and CR. Previous studies on multiple linear regression analysis also found that FT3 levels were affected by blood lipids (TC, HDL-C, and LDL-C) in T2DM patients. One of them showed that as FT3 levels increased, LDL-C levels also increased, which was the same as our results [18]. However, another study showed that as FT3 levels increased, TC levels decreased, which was contrary to our findings [7]. The reason for this discrepancy was that we considered the presence or absence of NAFLD, whereas the study by Wolide et al. did not include a subgroup analysis of NAFLD.

FT3 was significantly positively associated with NAFLD in T2DM patients (OR 1.367, 95% CI 1.068-1.751, *P* = 0.04), after adjusting for 28 biochemical indicators. But the mechanism of NAFLD remains uncertain. It has been proposed that interorgan crosstalk may contribute to the pathogenesis of NAFLD [19]. The core point is that the damage of the hypothalamic signaling pathway caused by factors such as inflammation and appetite leads to the development of obesity and NAFLD. The pituitary-hypothalamus-thyroid axis may also be affected, thereby affecting FT3 levels. There is also evidence that steatosis occurs during endoplasmic reticulum stress and subsequent production of reactive oxygen species (ROS), leading to the occurrence and progression of NAFLD [20]. The mechanism is that the signaling pathway is activated by disruption of endoplasmic reticulum homoeostasis, called unfolded protein response (UPR) [21].

Our study demonstrates that high level of FT3 may increase the risk of developing NAFLD in T2DM patients. In addition, as the FT3 tertile increases, the prevalence of NAFLD gradually increases (*P* for trend < 0.001). This is consistent with the previous results and further confirms our results. However, another point of view suggests that a low-normal FT3 is predictive of nonalcoholic steatohepatitis and advanced fibrosis [5, 22]. This inconsistent result is considered to be related to the heterogeneity of the study population, such as the use of hypoglycemic and lipid-lowering drugs, duration, and severity of NAFLD. What is special about this study is that patients with mild NAFLD account for 94% of all patients with NAFLD, and 97.2% of participants had FT3 levels within the normal reference range. In the study population of Manka et al., 54% of patients had mild NAFLD and the rest were patients with moderate to severe NAFLD [5, 22].

The current management of patients with T2DM and NAFLD is lifestyle intervention and oral hypoglycemic drugs such as metformin [4]. Finding various strategies to prevent and control NAFLD is very important. Researchers have explored the effects of Ramadan fasting on blood glucose, blood pressure, inflammation, and body composition in patients with NAFLD [23]. Studies have also shown that a low-carbohydrate and high-fat diet (LCHF) can reverse NAFLD and is beneficial for atherosclerotic dyslipidemia and insulin resistance [24]. In vitro and in vivo studies provide evidence of the potential utility of T3-dependent pathway activation in the treatment of NAFLD [25, 26]. Whether FT3 can be used as a drug for NAFLD still needs research to support it, especially in T2DM.

In conclusion, this study provides an independent positive association between FT3 and mild NAFLD among hospitalized T2DM patients. Whether FT3 is independently related to moderate and severe NAFLD still needs a lot of data to confirm.

## Figures and Tables

**Figure 1:** Flowchart of the study. NAFLD: nonalcoholic fatty liver disease. According to the inclusion criteria, a total of 77 people were excluded. Eventually, 859 patients were included in the research. Among them, 353 (41.1%) had T2DM with NAFLD and 506 (58.9%) had T2DM without NAFLD.

**Figure 2:** Instructions for using the nomogram.

**Figure 3:** Prevalence of NAFLD in three FT3 tertiles. FT3 tertiles (tertile 1: FT3 < 4.19; tertile 2: 4.19 ≤ FT3 < 4.87; and tertile 3: FT3 ≥ 4.87). As the FT3 tertile increases, the prevalence of NAFLD gradually increases (*P* for trend < 0.001). However, compared with tertile 1, tertile 2 (*P* = 0.026) and tertile 3 (*P* < 0.001) significantly increased the prevalence of NAFLD.

**Table 1:** Characteristics of hospitalized type 2 diabetes patients with or without NAFLD.

Variable	No NAFLD (*n* = 506)	NAFLD (*n* = 353)	Statistics	*P*
Age	51.41 ± 13.80	49.51 ± 12.22	0.989	*<*0.05
Gender				
M	319 (63.0)	217 (61.5)	0.219	0.64
W	187 (37.0)	136 (38.5)		
BMI	23.09 ± 3.30	26.23 ± 3.13	13.795	<0.001
AC (cm)	84.51 ± 9.40	92.13 ± 8.82	-11.75	<0.001
HC (cm)	91.79 ± 6.96	96.58 ± 7.01	-9.69	<0.001
SBP (mmHg)	132.18 ± 21.02	136.17 ± 19.30	-2.81	<0.001
DBP (mmHg)	77.97 ± 11.81	82.29 ± 12.56	-5.12	<0.001
T2DM duration (years)	56 (9)	3 (7)	-3.5	<0.001
Reason for hospitalization				
Abnormal blood glucose	264 (52.2)	214 (60.6)	7.87	<0.05
Diabetes complications	156 (30.8)	90 (25.5)		
Various local infections	53 (10.5)	36 (10.2)		
Other	33 (6.5)	13 (3.7)		
Occupation				
Blue collar	305 (60.3)	217 (61.5)	7.09	0.07
White collar	28 (5.5)	33 (9.3)		
Retirement	65 (12.9)	32 (9.1)		
Other	108 (21.3)	71 (20.1)		
Drinking history				
No	437 (98.0)	321 (99.4)	2.60	0.11
Abstaining from alcohol	9 (2.0)	2 (0.4)		
Smoking history				
No	373 (73.7)	271 (76.8)	0.45	0.92
Smoking occasionally	24 (4.7)	14 (4.0)		
Smoking regularly	45 (8.9)	34 (9.6)		
Abstaining from smoking	10 (2.0)	7 (2.0)		

BMI: body mass index; AC: abdominal circumference; HC: hip circumference; SBP: systolic blood pressure; DBP: diastolic blood pressure; M: man; W: woman. *P* < 0.05 was considered statistically significant.

**Table 2:** Biochemical indicators of hospitalized type 2 diabetes patients with or without NAFLD.

Variable	No NAFLD (*n* = 506)	NAFLD (*n* = 353)	Statistics (*Z*)	*P*
FINS (pmol/L)	53.93 (60.53)	73.91 (38.51)	-5.14	<0.001
FCP (nmol/L)	0.54 (0.63)	0.70 (0.47)	-7.17	<0.001
1h-CP (nmol/L)	1.07 (1.03)	1.33 (1.43)	-6.54	<0.001
2h-CP (nmol/L)	1.17 (1.23)	1.43 (1.87)	-5.76	<0.001
HbA1c (%)	8.70 (4.10)	8.30 (3.30)	-1.14	0.26
ABG (mmol/L)	12.70 (6.30)	12.10 (9.90)	-2.45	<0.001
FBG (mmol/L)	7.09 (3.46)	7.56 (4.28)	-2.22	<0.05
1hBG (mmol/L)	12.09 (4.07)	12.36 (4.48)	-4.38	<0.001
2hBG (mmol/L)	10.99 (5.62)	11.15 (4.80)	-3.38	<0.001
HOMA-IR	21.13 (24.05)	23.65 (14.29)	-4.99	<0.001
HOMA-*β*	294.88 (298.76)	257.52 (400.81)	-2.21	<0.05
TSH (mU/L)	1.77 (1.31)	1.60 (1.53)	-0.44	0.66
FT3 (pmol/L)	4.32 (0.89)	4.39 (0.58)	-4.07	<0.001
FT4 (pmol/L)	15.29 (3.03)	16.18 (3.35)	-0.76	0.45
ALT (U/L)	19.00 (15.20)	30.00 (22.00)	-6.87	<0.001
AST (U/L)	19.00 (10.00)	23.00 (10.50)	-3.84	<0.001
GGT (U/L)	24.00 (28.00)	33.00 (30.00)	-7.18	<0.001
UN (mmol/L)	4.78 (2.15)	4.64 (2.28)	-4.01	<0.001
CR (*μ*mol/L)	69.00 (39.00)	75.00 (39.00)	-2.33	<0.05
UA (*μ*mol/L)	342.00 (137.00)	372.00 (177.00)	-3.26	<0.001
TC (mmol/L)	1.72 (1.76)	2.12 (2.39)	-8.48	<0.001
TG (mmol/L)	4.33 (1.47)	4.68 (1.36)	-3.00	<0.01
HDL-C (mmol/L)	1.16 (0.39)	1.16 (0.29)	-1.10	0.27
LDL-C (mmol/L)	2.51 (1.01)	2.69 (1.02)	-1.33	0.18
24h-UTP (g/24 h)	91.60 (118.70)	82.20 (107.50)	-0.20	0.85
24hU-ABL (mg/24 h)	17.94 (47.43)	19.68 (22.59)	-0.84	0.4
24hU-ALB/CR (%)	18.31 (34.22)	15.43 (19.08)	-0.64	0.52
GFR (mL min^−1^ 1.73 m^−2^)	92.29 (49.98)	109.53 (53.11)	2.36	<0.05
DDi (ng/mL)	0.24 (0.26)	0.15 (0.22)	-5.21	<0.001
CRP (mg/L)	0.90 (4.50)	0.80 (4.20)	-1.42	0.16
HCY (*μ*mol/L)	10.10 (3.10)	10.90 (5.60)	-0.36	0.72

FINS: fasting insulin; FCP: fasting C peptide; ABG: admission blood glucose; FBG: fasting blood glucose; HbA1c: glycated hemoglobin; TSH: thyroid-stimulating hormone; FT3: free triiodothyronine; FT4: free four iodothyronine; ALT: alanine transferase; AST: aspartate aminotransferase; GGT: glutamyl transpeptidase; UN: urea nitrogen; CR: creatinine; UA: uric acid; TG: triglycerides; TC: total cholesterol; HDL: high-density lipoprotein cholesterol; LDL-C: low-density lipoprotein cholesterol; 24h-UTP: 24-hour urine protein quantification; 24hU-ABL: 24-hour urine albumin quantification; 24hU-ALB/CR: 24-hour urine albumin quantification to creatinine ratio; GFR: glomerular filtration rate; DDi: D-dimer; CRP: C-reactive protein; HCY: homocysteine; 1hBG: 1 h blood glucose; 1hINS: 1 h insulin; 1h-CP: 1 h C peptide; 2hBG: 2 h blood glucose; 2hINS: 2 h insulin; 2h-CP: 2 h C peptide; HOMA-IR: homeostasis model assessment-insulin resistance; HOMA-*β*: homeostasis model assessment-*β*.

**Table 3:** Pearson correlation analysis of parameters associated with FT3.

Variable	No NAFLD (*n* = 506)		NAFLD (*n* = 353)	
	*r*	*P*	*r*	*P*
Age	-0.148	<0.01	-0.342	<0.01
T2DM duration	-0.062	ns	-0.187	ns
BMI	0.057	ns	0.020	ns
SBP (mmHg)	0.025	ns	-0.560	ns
DBP (mmHg)	0.900	ns	0.690	ns
FINS (pmol/L)	-0.032	ns	-0.014	ns
FCP (nmol/L)	-0.049	ns	0.037	ns
2h-CP (nmol/L)	0.020	ns	0.056	ns
ABG (mmol/L)	-0.165	<0.01	-0.204	<0.01
FBG (mmol/L)	-0.099	<0.05	-0.069	ns
2hBG (mmol/L)	-0.019	ns	-0.083	ns
HbA1c	-0.128	<0.05	-0.173	<0.01
HOMA-IR	-0.026	ns	-0.049	ns
HOMA-*β*	-0.011	ns	0.036	ns
TSH (mU/L)	-0.139	<0.05	-0.125	<0.05
FT4 (pmol/L)	-0.019	ns	-0.058	ns
ALT (U/L)	0.023	ns	0.174	<0.01
AST (U/L)	-0.050	ns	0.013	ns
GGT (U/L)	-0.056	ns	0.089	ns
UN (mmol/L)	-0.105	<0.05	-0.117	<0.05
CR (*μ*mol/L)	-0.040	ns	-0.158	<0.01
UA (*μ*mol/L)	-0.058	ns	0.012	ns
TG (mmol/L)	-0.084	ns	0.007	ns
TC (mmol/L)	0.009	ns	0.062	ns
HDL-C (mmol/L)	-0.073	ns	-0.124	<0.05
LDL-C (mmol/L)	0.041	ns	0.202	<0.01
GFR (mL min^−1^ 1.73 m^−2^)	-0.400	ns	0.173	<0.01

BMI: body mass index; SBP: systolic blood pressure; DBP: diastolic blood pressure; FINS: fasting insulin; FCP: fasting C peptide; ABG: admission blood glucose; FBG: fasting blood glucose; HbA1c: glycated hemoglobin; TSH: thyroid-stimulating hormone; FT3: free triiodothyronine; FT4: free four iodothyronine; ALT: alanine transferase; AST: aspartate aminotransferase; GGT: glutamyl transpeptidase; UN: urea nitrogen; CR: creatinine; UA: uric acid; TG: triglycerides; TC: total cholesterol; HDL: high-density lipoprotein cholesterol; LDL-C: low-density lipoprotein cholesterol; GFR: glomerular filtration rate; CRP: C-reactive protein; 2hBG: 2 h blood glucose; 2hINS: 2 h insulin; 2h-CP, 2 h C peptide; HOMA-IR: homeostasis model assessment-insulin resistance; HOMA-*β*: homeostasis model assessment-*β*. *P* < 0.05 was considered statistically significant.

**Table 4:** Multiple linear regression analysis of parameters associated with FT3.

Variable	No NAFLD (*n* = 506)		NAFLD (*n* = 353)	
	*B*	*P*	*B*	*P*
Age	-0.016	<0.01	-0.023	<0.01
T2DM duration	/	/	/	/
BMI	0.03	<0.05	/	/
SBP (mmHg)	/	/	/	/
DBP (mmHg)	/	/	/	/
FINS (pmol/L)	/	/	/	/
FCP (nmol/L)	/	/	/	/
2h-CP (nmol/L)	/	/	/	/
ABG (mmol/L)	-0.039	<0.01	-0.300	<0.01
FBG (mmol/L)	/	/	/	/
2hBG (mmol/L)	/	/	/	/
HbA1c	-0.069	<0.01	-0.075	<0.01
HOMA-IR	/	/	/	/
HOMA-*β*	/	/	/	/
TSH (mU/L)	-0.020	<0.05	-0.022	<0.05
FT4 (pmol/L)	/	/	-0.028	<0.05
ALT (U/L)	/	/	0.006	<0.01
AST (U/L)	/	/	/	/
GGT (U/L)	/	/	0.003	<0.05
UN (mmol/L)	-0.041	<0.01	/	/
CR (*μ*mol/L)	/	/	-0.005	<0.01
UA (*μ*mol/L)	/	/	/	/
TG (mmol/L)	-0.006	<0.05	/	/
TC (mmol/L)	/	/	0.085	<0.05
HDL-C (mmol/L)	/	/	/	/
LDL-C (mmol/L)	0.090	<0.05	0.187	<0.01
GFR (mL min^−1^ 1.73 m^−2^)	/	/	/	/

BMI: body mass index; SBP: systolic blood pressure; DBP: diastolic blood pressure; FINS: fasting insulin; FCP: fasting C peptide; ABG: admission blood glucose; FBG: fasting blood glucose; HbA1c: glycated hemoglobin; TSH: thyroid-stimulating hormone; FT3: free triiodothyronine; FT4: free four iodothyronine; ALT: alanine transferase; AST: aspartate aminotransferase; GGT: glutamyl transpeptidase; UN: urea nitrogen; CR: creatinine; UA: uric acid; TG: triglycerides; TC: total cholesterol; HDL-C: high-density lipoprotein cholesterol; LDL-C: low-density lipoprotein cholesterol; GFR: glomerular filtration rate; CRP: C-reactive protein; 2hBG: 2 h blood glucose; 2hINS: 2 h insulin; 2h-CP: 2 h C peptide; HOMA-IR: homeostasis model assessment-insulin resistance; HOMA-*β*: homeostasis model assessment-*β*. *P* < 0.05 was considered statistically significant.

**Table 5:** Multivariate logistic regression analyses showing associations of NAFLD with FT3 among type 2 diabetic patients.

Model	FT3			
	*B*	*P*	OR	95% CI
Model 1	0.253	<0.05	1.288	1.062-1.562
Model 2	0.251	<0.05	1.286	1.006-1.644
Model 3	0.263	<0.05	1.301	1.028-1.645
Model 4	0.313	<0.05	1.367	1.068-1.751

Model 1 (adjusted for age, gender, T2DM duration, BMI, SBP, DBP, smoking history, TSH, and FT4), model 2 (adding FCP, 2h-CP, AbG, FbG, 2hbG, HOMA-IR, and HbA1c on the basis of model 1), model 3 (adding urea, CR, UA, and GFR to model 2), and model 4 (adding ALT, AST, GGT, TC, TG, HDL-C, and LDL-C to model 3). *P* < 0.05 was considered statistically significant.

## Data Availability

The data that support the findings of this study are available on request from the first author. The data are not publicly available due to privacy or ethical restrictions.

## Additional Points

*Strengths and Limitations of This Study*. (1) The advantage of this article is that the collected clinical data is more complete. (2) In this article, we control the effects of many variables on a nonalcoholic fatty liver. (3) The disadvantage is that the data in this study are cross-sectional data, which can only explain the correlation between indicators and facts, and they cannot determine their causal relationship.
